The article "6 month serologic response to the Pfizer-BioNTech COVID-19 vaccine among healthcare workers" was published in 2022. Journal: PLoS One.

# 6 month serologic response to the Pfizer-BioNTech COVID-19 vaccine among healthcare workers

**DOI:** 10.1371/journal.pone.0266781

**Published:** 2022-04-18

**Authors:** Jason Cham, Amitabh C. Pandey, Jacob New, Tridu Huynh, Lee Hong, Natalia Orendain, Eric J. Topol, Laura J. Nicholson

**Affiliations:** 1 Department of Medicine, Scripps Clinic/Scripps Green Hospital, La Jolla, California, United States of America; 2 Scripps Research Translational Institute, The Scripps Research Institute, La Jolla, California, United States of America; 3 Division of Cardiology, Scripps Clinic, La Jolla, California, United States of America; 4 Scripps Whittier Diabetes Institute, Scripps Hub Academic Research Core, La Jolla, California, United States of America; Qatar University, QATAR

## Abstract

**Aim:**

Healthcare workers (HCWs) were among the first group of people vaccinated with the Pfizer-BioNTech Covid-19 vaccine (BNT162b2). Characterization of the kinetics of antibody response to vaccination is important to devise future vaccination strategies. To better characterize the antibody response to BNT162b2, we analyzed the kinetics of IgG and IgM antibody response to 5 different SARS-CoV-2 epitopes over a period of 6 months.

**Methods and results:**

An observational single-centered study was conducted to evaluate the temporal dynamics of anti-SARS-CoV-2 antibodies following immunization with two doses of BNT162b2. Anti-SARS-CoV-2 antibodies were assessed using the Maverick SARS-CoV-2 multi-antigen panel (Genalyte Inc.). Healthcare workers aged ≥18 receiving BNT162b2 vaccination who self-reported no prior symptoms of COVID-19 nor prior COVID-19 PCR test positivity, were included in this study. HCWs developed an IgG antibody response to SARS-CoV-2 Spike S1, Spike S1 receptor binding domain (RBD), Spike S1S2 and Spike S2 after vaccination. IgG response was observed at two weeks following immunization in most participant samples and continued to increase at week 4, but subsequently decreased significantly starting at 3 months and up to 6 months. In contrast, IgM response to respective epitopes was minimal.

**Conclusion:**

Multiplex results demonstrate that, contrary to natural infection, immunization with BNT162b2 produces minimal anti-Spike IgM response. Polyclonal IgG response to Spike declined at 3 months and continued to do so up to 6 months.

## Introduction

The coronavirus disease 2019 (COVID-19) caused by SARS-CoV-2 infection was declared a pandemic by the World Health Organization on March 11, 2020. The Spike (S) protein receptor binding domain (RBD) on the surface of SARS-CoV-2 is critical for viral attachment, fusion and infection [1]. The Pfizer-BioNTech COVID-19 vaccine (BNT162b2) is a lipid-nanoparticle containing nucleoside-modified RNA encoding a secreted trimerized SARS-CoV-2 RBD and received FDA emergency use authorization on December 11, 2020 [2]. Among the first group of individuals to receive the vaccine were healthcare workers (HCWs). Recent studies on the antibody response to SARS-CoV-2 infection report robust humoral response including antiviral immunoglobulin-M (IgM), IgG, and IgA early after vaccination. The kinetics of producing these different antibody subtypes are variable [3–5]. We investigated the IgM and IgG antibody response to different S protein epitopes elicited by the BNT162b2 vaccine in HCWs sampled longitudinally for 6 months.

The article "6 month serologic response to the Pfizer-BioNTech COVID-19 vaccine among healthcare workers" was published in 2022. Journal: PLoS One.

## Materials and methods

### Study design

A single-centered observational study of HCWs designed to assess the temporal dynamics of anti-SARS-CoV-2 antibodies following immunization with BNT162b2 was conducted. Eligible participants were ≥18 years of age and worked at a large healthcare system. Participants were vaccinated with the Pfizer-BioNTech COVID-19 vaccine at week 0 (baseline) and week 3. Participant sera were collected at the following intervals: day of vaccination (baseline), week 2, week 4, 3 months, and 6 months. Samples were stored at -80 C until analysis.

### Serological assessment

Anti-SARS-CoV-2 antibodies were assessed using the Maverick SARS-CoV-2 multiantigen panel (Genalyte, Inc., San Diego, CA, USA), according to the manufacturer’s directions. This panel detects antibodies to five SARS-CoV-2 antigens: nucleocapsid, Spike S1 RBD, Spike S1S2, Spike S1, and Spike S2 based on photonic ring resonance. Briefly, 10 uL of each sample was added to the sample well plate array to assess baseline resonance. Subsequently, the samples were challenged over the respective antigens to assess specific IgM and IgG antibodies. Response measurements were reported in Genalyte response units (GRU). A proprietary machine learning algorithm was applied to generate a positive or negative call for response against the respective SARS-CoV-2 epitopes.

### Statistical analysis

The Friedman’s test was used to evaluate change in total antibodies, IgM, and IgG responses across all time points. Effect size was calculated via Kendall’s W coefficient. Pairwise comparisons between continuous variables were performed using the Wilcoxon rank sum test, followed by Bonferroni correction to address multiple testing. Statistical significance was set at p-value <0.05. All statistical analyses were performed with the statistical computing software R (https://www.r-project.org/).

### Ethics statement

This study was approved by the Scripps Health institutional review board, and all subjects provided written informed consent.

The article "6 month serologic response to the Pfizer-BioNTech COVID-19 vaccine among healthcare workers" was published in 2022. Journal: PLoS One.

## Results

### Study participant characteristics

17 participants were recruited to the study, of which 15 completed all five sera collections. Baseline characteristics of participants demonstrated an average age of 44 (29–57) years and 82% females. Of the 15 with complete data, there were 6 office staff, 3 nurses, 1 physician assistant, 2 medical assistants, 2 physicians, and 1 with unknown role. All participants self reported no prior symptoms of COVID-19 nor prior COVID-19 PCR test positivity.

### Serology results

Serologic response across time was significant for total antibody (χ2(49) = 485.99, p<0.0001), with a large effect size of 0.66. When examining IgG and IgM antibody responses separately, serologic response across time remained significant for both antibody groups (χ2(24) = 228.9, p<0.0001, and χ2(24) = 191.71, p<0.0001), respectively. The significant change in antibody response over time carried an effect size of 0.64 for IgG antibodies and 0.53 for IgM antibodies, suggesting that the observed significant serologic response over time is driven largely by IgG antibodies.

No participants demonstrated SARS-CoV-2 nucleocapsid IgM throughout the study period. One participant demonstrated SARS-CoV-2 nucleocapsid IgG, Spike S1 IgG and Spike S1 RBD IgG at the initial sera assessment, prior to immunization. While there was a significant change in the mean IgM response against most Spike epitopes between baseline and 6 months (Spike S1: 2.2 vs 1.2 GRU, p = 0.72; Spike S1 RBD: 25.7 vs 17.0 GRU, p = 0.045; Spike S1S2: 4.25 vs 2.73 GRU, p = 0.022; Spike S2: 7.73 vs 4.30 GRU, p = 0.001), overall IgM levels remained low at all time points (Fig 1).

**Fig 1:** Temporal IgM response to SARS-CoV-2 epitopes. IgM antibody response to respective SARS-CoV-2 epitopes at baseline, week 2, week 4, month 3 and month 6 in subjects administered Pfizer-BioNTech COVID-19 vaccine at week 0 and week 3. Antibody response is reported in Genalyte response units (GRU). NS represents a p-value >0.05, * represents a p-value ≤ 0.05, ** represents a p-value ≤ 0.01, *** represents a p-value ≤ 0.001, **** represents a p-value ≤ 0.0001.

Immunization resulted in an IgG predominant antibody response (Fig 2). IgG response was observed at two weeks following immunization in most subject samples. Furthermore, significant increases in mean response between baseline and week 4 were observed for anti-SARS-CoV-2 IgG against Spike S1 (26.9 vs 241 GRU, p = 0.00018), Spike S1 RBD (47.1 vs 289 GRU, p = 0.0018), Spike S1S2 (17.3 vs 81.9 GRU, p = 0.0015), and Spike S2 IgG (41.5 vs 152.1 GRU, p = 0.005). Subsequently, at 3 months and 6 months, there was a significant decrease in IgG response against all Spike domain epitopes (week 4 vs month 6 Spike S1: 241 vs 48.8 GRU, p = 0.00048; Spike S1 RBD: 289 vs 94.4 GRU, p = 0.00048; Spike S1S2: 81.9 vs 20.1 GRU, p = 0.00048; Spike S2: 152 vs 39.3 GRU, p = 0.00048).

The article "6 month serologic response to the Pfizer-BioNTech COVID-19 vaccine among healthcare workers" was published in 2022. Journal: PLoS One.

**Fig 2:** Temporal IgG response to SARS-CoV-2. IgG antibody response to respective SARS-CoV-2 epitopes at baseline, week 2, week 4, month 3 and month 6 in subjects administered Pfizer-BioNTech COVID-19 vaccine at week 0 and week 3. Antibody response is reported in Genalyte response units (GRU). NS represents a p-value >0.05, * represents a p-value ≤ 0.05, ** represents a p-value ≤ 0.01, *** represents a p-value ≤ 0.001, **** represents a p-value ≤ 0.0001.

## Discussion

In the present study, we examined the humoral response to the Pfizer-BioNTech COVID-19 vaccine by assaying 10 different immunoglobulins—IgM and IgG targeting each of 4 different Spike protein epitopes and 1 nucleocapsid epitope—against SARS-CoV-2. In natural infection, IgM and IgA have been reported present within five days of symptom onset and continue to be detected >21 days after symptom onset [3–5]. Antiviral IgG antibodies are detected about 10–14 days after symptom onset [2, 3]. We observed that, distinct from the early IgM response to natural infection, immunization with BNT162b2 produced a predominantly IgG polyclonal response, consistent with a recent study examining the serologic response to mRNA vaccination [6]. It has been hypothesized that the lipid component of the BNT162b2 vaccine formulation may drive the early IgG class switching [6]. One patient was found to have pre-existing IgG antibodies against the nucleocapsid consistent with prior infection. Upon follow-up, this patient reported a significant exposure to a symptomatic, PCR-positive individual, and thus is presumed to have had an asymptomatic infection. This further highlights the potential utility of a multiplex assay to distinguish between a vaccine response and a symptomatic or asymptomatic prior infection.

Estimates of mRNA vaccine efficacy among American HCWs during the period of December 2020 to March 2021, consistent with our study period, showed 90% efficacy against SARS-CoV-2 infection [7]. While the general population is starting to receive booster vaccinations against SARS-CoV-2, the duration of antibody response from mRNA vaccine remains uncertain. Antibody binding and neutralization response after the Moderna mRNA-1273 vaccination at 6 months have been reported to remain relatively high [8]. However, we found that the antibody response to the Spike protein significantly decreases at 6 months post vaccination with the Pfizer-BioNTech COVID-19 vaccine. This is in agreement with a recent study showing a decline of RBD-binding IgG and neutralizing antibodies [9]. Further studies should determine whether antibody decline correlates with waning immunity by examining the change in infection risk as time post-vaccination increases. Additionally, the cellular response should be evaluated to further define the complete landscape of vaccination-directed immunity. In the interim, this study provides additional data to inform ongoing investigations regarding the role of booster dosing to extend the level or duration of immunity, particularly in the context of emerging SARS-CoV-2 variants. Our study also provides information on anticipated response for future mRNA immunization targets and serves as a comparison for examination of humoral response in immunocompromised patients, a special population requiring innovative strategies to enhance vaccine immunogenicity.

The article "6 month serologic response to the Pfizer-BioNTech COVID-19 vaccine among healthcare workers" was published in 2022. Journal: PLoS One.

## Supporting information

S1 Table Raw Maverick SARS-CoV-2 multiantigen panel results. Raw values for IgM and IgG antibody response to respective SARS-CoV-2 epitopes at baseline, week 2, week 4, month 3 and month 6 in subjects administered Pfizer-BioNTech COVID-19 vaccine at week 0 and week 3. Antibody response is reported in Genalyte response units (GRU).
(XLSX)
